# Emodin protects against intestinal and lung injury induced by acute intestinal injury by modulating SP-A and TLR4/NF-κB pathway

**DOI:** 10.1042/BSR20201605

**Published:** 2020-09-24

**Authors:** Jingli Qian, Guoping Li, Xiaosheng Jin, Chunfang Ma, Wanru Cai, Na Jiang, Jisheng Zheng

**Affiliations:** 1 Department of Respiration, The Second Affiliated Hospital of Zhejiang Chinese Medical University, Hangzhou 310005, Zhejiang, China; 2 Department of Respiration, Tongde Hospital of Zhejiang Province, Hangzhou 310012, Zhejiang, China; 3 Clinical Laboratory, Zhejiang Provincial People’s Hospital, Hangzhou 310014, Zhejiang, China

**Keywords:** acute intestinal injury, emodin, lung injury, surfactant protein-A, toll-like receptor 4

## Abstract

**Objective:** Our aim was to investigate the effect of emodin on intestinal and lung injury induced by acute intestinal injury in rats and explore potential molecular mechanisms.

**Methods:** Healthy male Sprague–Dawley (SD) rats were randomly divided into five groups (*n*=10, each group): normal group; saline group; acute intestinal injury model group; model + emodin group; model+NF-κB inhibitor pynolidine dithiocarbamate (PDTC) group. Histopathological changes in intestine/lung tissues were observed by Hematoxylin and Eosin (H&E) and terminal deoxynucleotidyl transferase biotin-dUTP nick-end labeling (TUNEL) staining. Serum IKBα, p-IKBα, surfactant protein-A (SP-A) and toll-like receptor 4 (TLR4) levels were examined using enzyme-linked immunosorbent assay (ELISA). RT-qPCR was performed to detect the mRNA expression levels of IKBα, SP-A and TLR4 in intestine/lung tissues. Furthermore, the protein expression levels of IKBα, p-IKBα, SP-A and TLR4 were detected by Western blot.

**Results:** The pathological injury of intestinal/lung tissues was remarkedly ameliorated in models treated with emodin and PDTC. Furthermore, the intestinal/lung injury scores were significantly decreased after emodin or PDTC treatment. TUNEL results showed that both emodin and PDTC treatment distinctly attenuated the apoptosis of intestine/lung tissues induced by acute intestinal injury. At the mRNA level, emodin significantly increased the expression levels of SP-A and decreased the expression levels of IKBα and TLR4 in intestine/lung tissues. According to ELISA and Western blot, emodin remarkedly inhibited the expression of p-IKBα protein and elevated the expression of SP-A and TLR4 in serum and intestine/lung tissues induced by acute intestinal injury.

**Conclusion:** Our findings suggested that emodin could protect against intestinal and lung injury induced by acute intestinal injury by modulating SP-A and TLR4/NF-κB pathway.

## Introduction

Acute intestinal injury is a serious but common clinical event, based on the pathological basis of ischemic edema of the intestinal wall and increased permeability of the intestinal mucosa, with or without intra-abdominal hypertension syndrome [1]. Studies have confirmed that acute intestinal injury can be caused by a variety of factors (such as trauma, shock, severe infection, sepsis, and excessive fluid resuscitation). If the ischemic edema is not corrected in time, the permeability of the intestinal mucosa would further increase, eventually leading to acute intestinal injury syndrome or even multiple organ dysfunction syndrome (MODS) [2,3]. It has been confirmed that lung is the most vulnerably affected organs by MODS, with a high mortality, of approximately 40% [4–6]. However, there is currently no effective medical treatment.

Emodin is one of the effective ingredients of rhubarb, which belongs to the class of hydroxyanthraquinones [7–9]. Its chemical structure is 1,3,8-trihydroxy-6methylanthraquinone (1,3,8-trihydroxy-6methy lanthraquinone). Increasing research has confirmed that emodin can improve intestinal blood circulation, promote intestinal motility, stimulate intestinal secretion, kill microorganisms, reduce intestinal mucosal permeability, anti-inflammatory and immune regulation [10]. Studies have confirmed that emodin has a protective effect on intestinal mucosal barrier damage caused by various risk factors [11]. Moreover, emodin can protect the tight junction structure and reduce damage and inhibit the apoptosis of intestinal mucosa cells [12–14].

It has been reported that several signaling pathways are involved in the development of intestinal and lung injury induced by acute intestinal injury such as surfactant protein-A (SP-A) [15] and toll-like receptor 4 (TLR4)/NF-κB [16]. SP-A is a multimeric protein in the airways and alveoli of the lungs [17]. TLRs are cell transmembrane receptors and pathogenic pattern recognition receptors in the innate immune system [18–20]. Thus, targeting these signaling pathways could become a potential treatment strategy. In the present study, we hypothesized that emodin could protect against intestinal and lung injury induced by acute intestinal injury. In-depth research found that emodin could mediate SP-A and TLR4/NF-κB activation against intestinal and lung injury for acute intestinal injury rats.

## Materials and methods

### Animals

A total of 40 healthy male Sprague–Dawley (SD) rats (2 months old; weighing 250 ± 30 g) were purchased from Shanghai Experimental Animal Center, Chinese Academy of Sciences. All rats were housed at 21 ± 1°C with 40–70% humidity and a 12-h light/dark cycle. Animal experiments were carried out in the Laboratory of Tongde Hospital of Zhejiang Province. This experiment was presented in strict accordance with the recommendations in the Guide for the Care and Use of Laboratory Animals of the National Institutes of Health. The study was approved by the ethical committee of Tongde Hospital of Zhejiang Province (2019014).

### Experimental groups

All rats were randomly divided into five groups (*n*=10, each group): normal group; saline group; acute intestinal injury model group; acute intestinal injury model + emodin group; acute intestinal injury model + pynolidine dithiocarbamate (PDTC) group.

### Acute intestinal injury model

In the present study, 3% acetic acid was injected into the colon to establish a rat model of acute intestinal injury. In brief, after intraperitoneal injection of 50 mg/kg pentobarbital sodium, the rats were turned upside down. For the rats in the acute intestinal injury model group, intestinal injury model + emodin group and intestinal injury model + PDTC group, 15 ml/kg of 3% acetic acid was slowly infused into the colon approximately 5 cm from the anus; rats in the saline group were infused with an equal amount of saline. After infusion, the rats were inverted for 3 min to distribute the drug evenly on the colorectal wall. Rats in the normal group did not receive any treatment. Twelve hours before modeling, rats in saline group and acute intestinal injury model group were pretreated with 5 ml/kg saline intraperitoneally; rats in intestinal injury model + emodin group were pretreated with 5 ml/kg emodin solution intraperitoneally. At 12 and 24 h after modeling, rats in saline group and acute intestinal injury model group were intraperitoneally injected with 5 ml/kg saline; rats in intestinal injury model + emodin group were intraperitoneally injected with 5 ml/kg emodin solution. Rats in intestinal injury model + PDTC group were injected intraperitoneally with 5 ml/kg saline at 12 h before modeling, 12 and 24 h after modeling and were intraperitoneally injected with 20 ml/kg PDTC at 1 h before modeling. The preparation method of emodin solution was as follows: emodin 100 mg was dissolved in 20 ml of 0.1% NaOH solution (to make a concentration of 5 g/l). The PDTC solution preparation method was as follows: 100 mg PDTC was dissolved in 20 ml of 20% dimethyl sulfoxide (DMSO; to make a concentration of 5 g/l). After 36 h of modeling, the rats were killed with an overdose of 50 mg/kg pentobarbital sodium by intraperitoneal injection. The large intestine tissues approximately 2 cm from the upper anus 4–6 cm and the left lower lobe of the lung tissues were removed and fixed with 10% formaldehyde for Hematoxylin and Eosin (H&E) staining. The large intestine tissues approximately 6–8 cm above the anus and the right lower lobe of the lung tissues were removed, rinsed with PBS for 1–2 min, and stored at −70°C.

### Histological analysis

Fresh tissues were fixed in 4% paraformaldehyde (E672002, Sangon Biotech, Shanghai, China) for 24 h. After dehydration and paraffin embedding, the tissues were cut into 4-μm-thick sections. Following dewaxing to water, the sections were stained with Harris Hematoxylin for 5–10 min and Eosin dye solution for 1–3 min. After dehydration and sealing, the pathological changes were observed under an optical microscope (Olympus, Japan). The severity of intestinal injury and lung injury was assessed according to Nadler and Szapiel scoring systems, respectively. Apoptosis was detected using terminal deoxynucleotidyl transferase biotin-dUTP nick-end labeling (TUNEL) apoptosis detection kit (ATK00001, Pujian Biotechnology Co., Ltd., Wuhan, China) according to the manufacturer’s instructions.

### Enzyme-linked immunosorbent assay

Serum was naturally coagulated at room temperature for 30 min. After centrifugation at 1000×***g*** for approximately 20 min, the supernatant was harvested. Rat IKBα ELISA kit (OM626522, OmnimAbs, Shanghai, China), rat p-IKBα ELISA kit (OM626523, OmnimAbs), rat SP-A ELISA kit (OM626521, OmnimAbs), rat TLR4 ELISA kit (OM589197, OmnimAbs) were used for enzyme-linked immunosorbent assay (ELISA) according to the manufacturer’s protocols. Absorbance at 450 nm was measured using automatic microplate reader (Thermo Scientific).

### RT-qPCR

Tissues were lysed using TRIzol™ Reagent (15596018, Invitrogen, Carlsbad, California, U.S.A.) at room temperature for 5 min. After centrifugation at 12000 rpm at 4°C, supernatant was harvested. Total RNA was then extracted. Purity and concentration of 1 μl RNA was determined according to OD260/OD280 using UV spectrophotometer. Then, RNA was reverse transcribed into cDNA. The reverse transcription system was composed of 1 μl primescript enzyme mix, 1 μl RT primer mix, 4 μl of 5× primescript buffer, 2.9148 μg RNA and 20 μl RNase-free H_2_O. The reaction procedure was as follows: 37°C for 15 min, 85°C for 5 s and 4°C hold. The expression levels of genes were examined using RT-qPCR according to the following reaction procedure: 95°C for 10 min; 40 cycles of 95°C for 10 s, 60°C for 15 s and 72°C for 20 s; 65–95°C, 0.5°C/5 s. GAPDH served as a housekeeping gene. The relative expression levels were calculated with the 2^−ΔΔ*C*_t_^ method. The primer sequences are listed in Table 1.

**Table 1:** Primer sequence information for RT-qPCR

Gene name	5′–3′sequence	Product size
*IκBα*	5′-TTGACTCAGACCTGTACGCC-3′ (forward)	231 bp
	5′-ACACTTCAACAGGAGCGAGA-3′ (reverse)	
*SP-A*	5′-CAAGGGAGAGCCTGGAGAAA-3′ (forward)	181 bp
	5′-GTTGACTGACTGCCCATTGG-3′ (reverse)	
*TLR4*	5′-TATCGGTGGTCAGTGTGCTT-3′ (forward)	167 bp
	5′-CTCGTTTCTCACCCAGTCCT-3′ (reverse)	
*GAPDH*	5′-ACTCCCATTCTTCCACCTTTG-3′ (forward)	105 bp
	5′-CCCTGTTGCTGTAGCCATATT-3′ (reverse)	

### Western blot

Tissue samples were lysed using RIPA lysis buffer (P0013B, Beyotime, Beijing, China), followed by 140000×***g*** centrifugation at 4°C for 15 min on the ice. Then, supernatant was collected. The concentration of extracted protein was determined using BCA protein quantitative detection kit (P0009, Beyotime). Protein samples were subjected on to SDS/PAGE and transferred to PVDF membrane. After that, membrane was blocked using 5% milk/TBST at room temperature for 1 h. Membrane was incubated with 30 μg primary antibodies against SP-A (1:1000; ab51891, Abcam, Cambridge, U.K.), IKBα (1:1500; 10268-1-AP, Proteintech, Chicago, U.S.A.), p-IKBα (1:1000; AP0707, ABclonal, Wuhan, China), TLR4 (1:600; BS3489, Bioworld, Minnesota, U.S.A.) and GAPDH (1:5000, SA00001-2, Proteintech, Wuhan, China) at 4°C overnight, followed by incubation with horseradish peroxidase-labeled goat anti-rabbit secondary antibody (1:5000, ab150077, Abcam) and goat anti-rat secondary antibody (1:5000, ab150165, Abcam) at room temperature for 1 h. Protein blots were visualized using Enhanced Luminol reagent and oxidizing reagent. The results were observed using ChemiDoc™ XRS+ Gel imaging system (Bio-Rad, Shanghai, China).

### Statistical analysis

All statistical analysis was carried out using GraphPad Prism 8.0 (GraphPad Software, San Diego, CA, U.S.A.). Each experiment was repeated at least three times. Data were expressed as mean ± standard deviation (SD). Multiple comparisons were performed by one-way ANOVA test. *P*<0.05 was considered statistically significant.

## Results

### Emodin could ameliorate intestinal injury in rats with acute intestinal injury

H&E staining results showed that, for rats in the normal group, the intestinal tissue structure was complete, the chorionic glands were arranged regularly, the mucosal layer, submucosa and lamina propria were intact. No obvious edema and tissue lesions were found (Figure 1A). The intestinal structure of the rats in the saline group was normal, with occasional slight mucosal epithelial spotting (Figure 1A). The intestinal lesions of rats in the model group were obvious, and some intestinal villi were necrotic and shed or even disappeared. The submucosal muscle layer was broken, the lamina propria was necrotic, severe bleeding was accompanied by a large number of inflammatory cell infiltration (Figure 1A). The pathological damage of intestine of acute intestinal injury rats treated with emodin was significantly lighter than that in the model group. Some intestinal villi were necrotic and shed, and the lamina edema was accompanied by local bleeding and inflammatory cell infiltration (Figure 1A). In the PTDC + model group, the degree of pathological damage was significantly lighter than that in the model group. Only some intestinal villi were necrotic and shed, and the lamina propria was accompanied by local bleeding and inflammatory cell infiltration (Figure 1A). The pathological injury of the intestine was evaluated according to the Nadler scoring system. The Nadler scores of model group were significantly higher than of saline group. After treatment with emodin or PDTC, the Nadler scores were distinctly decreased (Figure 1B). However, there was no statistical significance between model + emodin group and model + PDTC group.

**Figure 1:** Emodin could ameliorate intestinal injury in rats with acute intestinal injury (**A**) Representative images of intestinal tissues of H&E staining results. Magnification: 10×, 20× and 40×. (**B**) Intestinal injury assessment according to Nadler score system. PDTC or emodin significantly decreased the intestinal injury score of acute intestinal injury rats. All mice were randomly divided into five groups: normal group; saline group; acute intestinal injury model group; intestinal injury model + emodin group; intestinal injury model + PDTC group. *P<0.05; **P<0.01; ****P<0.0001; ns, no statistical significance.

### Emodin improves lung injury in rats with acute intestinal injury

In the normal group and saline group, the lung tissue structure was clear, the alveolar wall was thin, the capillary wall was intact, and inflammatory cells exuded occasionally (Figure 2A). In the acute intestinal injury model group, the exudate of alveolar inflammatory cells increased, the alveolar wall thickened, pulmonary interstitial edema and congestion was found in the alveolar cavity, capillary dilation was found in the pulmonary interstitial, and occasionally cellulose-like exudates (Figure 2A). The lung injury in the model + emodin group and model + PTDC group was significantly lighter than the model group. The lung tissue structure was clearer, the alveolar wall became thinner, and fewer inflammatory cells exuded (Figure 2A). According to the Szapiel score classification, the severity of lung injury in the model group was obviously higher than in saline group (Figure 2B). However, emodin and PDTC treatment remarkedly ameliorated the severity of lung injury of rats with acute intestinal injury (Figure 2B). No statistical significance was found between model + emodin group and model + PDTC group.

**Figure 2:** Emodin improves lung injury in rats with acute intestinal injury (**A**) Representative images of lung tissues of H&E staining results. Magnification: 10×, 20× and 40×. (**B**) Intestinal injury assessment according to Szapiel score classification. PDTC or Emodin distinctly suppressed the lung injury score of acute intestinal injury rats. All mice were randomly divided into five groups: normal group; saline group; acute intestinal injury model group; intestinal injury model + emodin group; intestinal injury model + PDTC group. *P<0.05; **P<0.01; ***P<0.001; ns, no statistical significance.

### Emodin protects intestinal cells against apoptosis in rats with acute intestinal injury

To observe the effect of emodin on intestinal cell apoptosis in rats with acute intestinal injury, TUNEL assay was conducted (Figure 3A). As expected, the apoptosis levels of intestinal cells in rats with acute intestinal injury were significantly higher than in saline group (Figure 3B). After treatment with emodin and PDTC, the apoptosis levels of intestinal cells in rats with acute intestinal injury were distinctly improved (Figure 3B).

**Figure 3:** Emodin protects intestinal cells against apoptosis in rats with acute intestinal injury (**A**) Representative images of intestinal tissues for TUNEL assay results. Magnification: 200×. Bar value: 50 μm. (**B**) Relative apoptosis levels were determined in intestinal tissues. PDTC or Emodin significantly inhibited the apoptosis levels of intestinal tissues in the acute intestinal injury models. *P<0.05; **P<0.01; ***P<0.001; ns, no statistical significance.

### Emodin decreases apoptosis in the lung cells in rats with acute intestinal injury

We also investigated the effects of emodin on apoptosis of lung cells in rats with acute intestinal injury using TUNEL assay (Figure 4A). Similar to intestinal cells, the apoptosis levels of lung cells in model group was remarkedly increased compared with saline group (Figure 4B). Moreover, emodin and PDTC treatment distinctly ameliorated the apoptosis levels of lung cells in rats with acute intestinal injury (Figure 4B).

**Figure 4:** Emodin decreases apoptosis in the lung cells in rats with acute intestinal injury (**A**) Representative images of lung tissues for TUNEL assay results. Magnification: 200×. Bar value: 50 μm. (**B**) Relative apoptosis levels were quantified in lung tissues. PDTC or emodin significantly inhibited the apoptosis levels of lung tissues in the acute intestinal injury models. *P<0.05; **P<0.01; ns, no statistical significance.

### Emodin ameliorates the levels of p-IKBα, SP-A and TLR4 in serum of rats with acute intestinal injury

ELISA results showed that, no obvious changes in IKBα levels occurred in serum of rats with acute intestinal injury (Figure 5A). However, p-IKBα levels were significantly increased in serum of rats with acute intestinal injury compared with saline group (Figure 5B). Both emodin and PDTC treatment could distinctly decrease the levels of p-IKBα in serum of rats with acute intestinal injury (Figure 5B). Intriguingly, the inhibitory effects of emodin on p-IKBα levels were significantly higher than PDTC in serum of rats with acute intestinal injury (Figure 5B). Also, the levels of SP-A were remarkedly decreased in serum of rats with acute intestinal injury compared with saline group (Figure 5C). After treatment with emodin or PDTC, the serum levels of SP-A were significantly increased in rats with acute intestinal injury (Figure 5C). Furthermore, we found that the serum levels of SP-A in model + emodin group were significantly higher than in model + PDTC group (Figure 5C). We also examined the serum levels of TLR4 in rats with acute intestinal injury. Compared with saline group, the serum levels of TLR4 were significantly lower in model group (Figure 5D). Both emodin and PDTC treatment remarkedly elevated the serum of TLR4 in rats with acute intestinal injury (Figure 5D). However, there was no statistical significance between emodin and PDTC treatment.

**Figure 5:** ELISA results showed that emodin could ameliorate the levels of p-IKBα, SP-A and TLR4 in the serum of rats with acute intestinal injury (**A**) IKBα; (**B**) p-IKBα; (**C**) SP-A; (**D**) TLR4. **P<0.01; ***P<0.001; ****P<0.0001; ns, no statistical significance.

### Emodin could mediate the expression levels of p-IKBα, SP-A and TLR4 in intestinal tissues in rats with acute intestinal injury

RT-qPCR results showed that the mRNA expression levels of SP-A in intestinal tissues of rats with acute intestinal injury were significantly lower compared with saline group (Figure 6A). We found that emodin not PDTC treatment distinctly elevated the mRNA expression levels of SP-A (Figure 6A). Furthermore, IKBα and TLR4 mRNA levels had significantly higher expression levels in intestinal tissues of rats with acute intestinal injury than in saline group (Figure 6B,C). However, both emodin and PDTC treatment could elevate the mRNA expression levels of IKBα and TLR4 (Figure 6B,C). We also conducted Western blot assays (Figure 6D). Consistent with RT-qPCR assay results, low SP-A protein levels were found in intestinal tissues of rats with acute intestinal injury, which were significantly ameliorated by emodin treatment not PDTC treatment (Figure 6E). No significant changes in IKBα protein expression were found in intestinal tissues of rats with acute intestinal injury (Figure 6F). However, p-IKBα and TLR4 protein expression levels were significantly elevated in model group than in saline group (Figure 6G,H). Also, both emodin and PDTC treatment could decrease the expression levels of p-IKBα and TLR4 proteins (Figure 6G,H).

**Figure 6:** Emodin could mediate the expression levels of p-IKBα, SP-A and TLR4 in the intestinal tissues of rats with acute intestinal injury RT-qPCR results showed the mRNA expression levels of SP-A (**A**), IKBα (**B**) and TLR4 (**C**) in intestinal tissues. (**D**) Representative images of Western blot. The expression levels of SP-A (**E**), IKBα (**F**), IKBα (**G**) and TLR4 (**H**) proteins were quantified in intestinal tissues according to the Western blot results. *P<0.05; **P<0.01; ***P<0.001; ****P<0.0001; ns, no statistical significance.

### Emodin could regulate the expression levels of p-IKBα, SP-A and TLR4 in lung tissues induced by acute intestinal injury

We also detected the mRNA expression levels of SP-A, IKBα and TLR4 in lung tissues in rats with acute intestinal injury. As shown in Figure 7A, the expression levels of SP-A mRNA were significantly lower in lung tissues of rats in model groups compared with saline group. Emodin could obviously ameliorate the expression levels of SP-A in lung tissues of rats with acute intestinal injury. Moreover, emodin not PDTC treatment significantly decreased the mRNA expression levels in lung tissues of rats with acute intestinal injury (Figure 7B). TLR4 had a higher mRNA level in lung tissues of rats with acute intestinal injury compared with saline group, which was significantly decreased by emodin and PDTC treatment (Figure 7C). Western blot was then performed (Figure 7D). Emodin treatment distinctly increased the protein levels of SP-A in lung tissues induced by acute intestinal injury (Figure 7E). Similarly, no significant changes in IKBα protein were found in lung tissues induced by acute intestinal injury (Figure 7F). Furthermore, emodin and PDTC treatment remarkedly decreased the expression levels of p-IKBα and TLR4 proteins in lung tissues induced by acute intestinal injury (Figure 7G,H).

**Figure 7:** Emodin could regulate the expression levels of p-IKBα, SP-A and TLR4 in lung tissues induced by acute intestinal injury RT-qPCR results showed the mRNA expression levels of SP-A (**A**), IKBα (**B**) and TLR4 (**C**) in the lung tissues. (**D**) Representative images of Western blot. The expression levels of SP-A (**E**), IKBα (**F**), IKBα (**G**) and TLR4 (**H**) proteins were quantified in the lung tissues based on the Western blot results. *P<0.05; **P<0.01; ***P<0.001; ****P<0.0001; ns, no statistical significance.

## Discussion

Our results showed that emodin could ameliorate the intestinal and lung injury induced by acute intestinal injury in rats. Furthermore, TUNEL assay results showed that emodin could improve the apoptosis of intestinal and lung tissues in rats with acute intestinal injury. Mechanically, emodin could protect against intestinal and lung injury induced by acute intestinal injury in rats via SP-A and TLR4/NF-κB pathway.

TLRs play an important role in the regulation of phagocytosis of acute inflammatory response cells [21], cell signaling [22] and apoptosis [23]. Among all TLRs, the ligand of TLR4 is lipopolysaccharide, a cell wall component of Gram-negative bacteria. It has been confirmed that TLR4 is closely related to acute intestinal injury and intestinal infection [24]. Consistent with previous studies, in our study, we found that TLR4 levels were remarkedly decreased in serum, intestinal and lung tissues of rats with acute intestinal injury, which were ameliorated by emodin treatment. TLR4/NF-κB pathway has been reported to be closely related to acute intestinal/lung injury [2,25,26]. The NF-κB family consists of five members: P50, P52, p65/RelA, RelB and c-Rel. These members exist in the cytoplasm in the form of inactive dimers in combination with the NF-κB inhibitor IκB [27]. The activated NF-κB is quickly transferred to the nucleus and mediates gene transduction including various factors. Three members of the IκB family have been discovered, including IκBα, IκBβ and IκBε. Among them, the phosphorylation of IκBα is the fastest, thus, its phosphorylation (p-IκBα) is regarded as a sign of NF-κB activation [28]. In this study, p-IκBα levels were significantly elevated in serum, intestinal and lung tissues of rats with acute intestinal injury, indicating that NF-κB could be activated. PDTC is a specific inhibitor of NF-κB, which mainly inhibits the activity of NF-κB by reducing the nuclear translocation of NF-κB [29]. Our results showed that PDTC treatment could reduce the p-IκBα levels in serum, intestinal and lung tissues of rats with acute intestinal injury, suggesting that NF-κB activation was inhibited.

SP-A is a member of the protein collectin family, characterized by a collagen-like region at the NH_2_ end and a lectin domain at the COOH end. SP-A can regulate the lung immune response [30–32]. By combining with various pathogens, SP-A can enhance the absorption of pathogens by phagocytes [33]. Moreover, SP-A can significantly reduce intestinal mucosal damage, apoptosis and inflammation [15]. Thus, in this study, we detected SP-A expression in the intestinal and lung tissues. As expected, it was found that SP-A was lowly expressed in the intestinal and lung tissues of model rats. In the acute intestinal injury model group, SP-A expression was distinctly decreased in the serum, intestine and lung tissues, while p-IκBα and TLR4 expression increased. Emodin or PDTC treatment reversed the expression of the above components. Thus, emodin could mediate SP-A and TLR4/NF-κB pathway in serum, intestine and lung tissues of rats with acute intestinal injury.

## Conclusion

In the present study, our results suggested that emodin could protect against intestinal and lung injury induced by acute intestinal injury in rats via SP-A and TLR4/NF-κB pathway. Thus, emodin could become a potential drug for treatment of acute intestinal/lung injury, which is worth further exploration.

## Data Availability

The datasets analyzed during the current study are available from the corresponding author on reasonable request.

## Abbreviations

ELISA: enzyme-linked immunosorbent assay
H&E: Hematoxylin and Eosin
MODS: multiple organ dysfunction syndrome
PDTC: pynolidine dithiocarbamate
SP-A: surfactant protein-A
TLR4: toll-like receptor 4
TUNEL: terminal deoxynucleotidyl transferase biotin-dUTP nick-end labeling
